# Pharmacokinetics and Toxicokinetics of Artemisinin-Hydroxychloroquine Sulfate Tablets in Rats and Dogs

**DOI:** 10.1155/2021/6830459

**Published:** 2021-10-21

**Authors:** Xiaobo Li, Jiaoting Hu, Yueming Yuan, Yunhan Wang, Zheng Yuan, Ruidong Liu, Shouya Zhang, Zhiyong Xu, Qi Wang, Qin Xu, Li Ru, Jianping Song

**Affiliations:** ^1^Artemisinin Research Center, Guangzhou University of Chinese Medicine, Guangzhou 510405, China; ^2^Sci-Tech Industrial Park, Guangzhou University of Chinese Medicine, Guangzhou 510445, China; ^3^The First Affiliated Hospital of Guangzhou University of Chinese Medicine, Guangzhou 510405, China

## Abstract

Artemisinin-hydroxychloroquine sulfate tablets (AH) are relatively inexpensive and a novel combination therapy for the treatment of all forms of malaria, especially aminoquinine drug-resistant strains of *P. falciparum*. Our aim was to assess the pharmacokinetics (PK) and toxicokinetics (TK) of AH following oral administration in Sprague Dawley rats and Beagle dogs by using the liquid chromatography tandem mass spectrometry methods (LC-MS/MS). The PK studies were carried out in eighteen rats at three doses and six dogs at three rounds of three doses after a single oral administration of AH. The TK studies in rats and dogs were accompanied by the 14-day repeated dosing studies. The PK results revealed that artemisinin was absorbed and cleared rapidly in rats with obvious gender difference and interindividual variability, and the systemic exposure with regard to AUC was positively correlated with the dosage in female rats. However, the kinetics parameters of artemisinin in dogs were not obtained because the plasma concentration was undetectable. The absorption and elimination of hydroxychloroquine in dogs and rats were relatively slow, and no gender difference was observed. The AUC of hydroxychloroquine showed a linear correlation with the dosage, but *C*_max_ varied significantly among individuals. After 14-day repeated oral administration of AH, hydroxychloroquine shows an increase in systemic exposure and accumulation in rats and dogs, whereas the AUC and *C*_max_ of artemisinin remarkably decreased in female rats due to its autoinduction metabolism. The TK results were basically consistent with the dose- and time-dependent toxic reaction in 14-day repeated dosing studies of AH in rats and dogs. The information from our studies could be helpful for further pharmacological and toxicological research and clinical application of AH.

## 1. Introduction

Malaria, caused by *Plasmodium*, is one of the most prevalent vector-borne diseases in the world. According to the report of the World Health Organization (WHO), about 3.2 billion people (nearly half of the world's population) globally are at risk of malaria. It is estimated that 229 million cases of malaria occurred worldwide in 2019, leading to 409,000 malaria deaths [1]. Malaria is not only a serious health problem in developing countries, but also a social problem that hinders economic development and social progress. Artemisinin-based combination therapies (ACTs), combining an artemisinin or its derivatives with a partner drug, are recommended by the WHO as the first-line treatment for uncomplicated *Plasmodium falciparum* malaria. The role of the artemisinin compound is to reduce the number of parasites during the first three days of treatment (reduction of parasite biomass), while the role of the partner drug is to eliminate the remaining parasites (cure). Drugs compatible with artemisinins, such as piperquine phosphate, pyrimethamine, mefloquine, and amodiaquine, are widely used in the treatment of malaria but have developed resistance [2, 3]. Although artemisinin and its derivatives also have drug resistance in the Cambodia-Thailand border area [4, 5], they remain available as long as the collocation drugs in ACTs are effective locally. ACTs are still effective in most cases. In this regard, we hope to choose an antimalarial drug that is not widely used and is compatible with artemisinin to form a new and effective compound, which has broad application prospects.

Hydroxychloroquine sulfate is a derivative of chloroquine, which belongs to the 4-aminoquinolines and has similar effects to chloroquine, such as malaria treatment, immune regulation, antibacterial, and so on [6]. However, some adverse drug reactions of hydroxychloroquine sulfate may occur in clinical applications, including retinopathy, cardiomyopathy, neuromuscular disease, and myopathy [7]. The clinical application of chloroquine is limited because of its serious drug resistance and side effects [8]. Hydroxychloroquine is relatively less toxic and has been currently used for rheumatoid arthritis, but it is being rarely used clinically as an antimalarial drug [9, 10]. Recently, we have developed a compound preparation composed of artemisinin and hydroxychloroquine sulfate (AH) for the treatment of malaria. Our previous studies have demonstrated that the combination of artemisinin and hydroxychloroquine sulfate can improve the therapeutic effect of malaria, decrease the dose of both, reduce the toxic side effects of hydroxychloroquine, and postpone the progress of single drug resistance (unpublished data). Thus, we have applied for a patent for this compound, which is not only used to treat malaria, but may also be used to treat immune diseases in the future.

The current study has been undertaken to generate pharmacokinetic and toxicokinetic data for AH following oral administration in Sprague Dawley (SD) rats and Beagle dogs, which are the rodents and nonrodents conventionally used in preclinical studies. The scientific information obtained from these studies would be taken into consideration for safety evaluation and clinical application of AH.

## 2. Materials and Methods

### 2.1. Chemicals and Reagents

Artemisinin-hydroxychloroquine sulfate tablets (AH, lot # 20170901) were produced in a GMP facility of Artepharm Co. Ltd (Meizhou, China). Each tablet (235 mg) contains artemisinin (50 mg) and hydroxychloroquine sulfate 64.6 mg). Artemisinin (C_15_H_22_O_5_, purity 99.6%) was purchased from the National Institute for Food and Drug Control (Beijing, China). Hydroxychloroquine sulfate (C_18_H_28_ClN_3_O_5_S, purity 98%) was purchased from Shanghai yuanye Bio-Technology Co. Ltd (Shanghai, China). Hydroxychloroquine-d4 sulfate (C_18_H_24_D_4_ClN_3_O_5_S, purity 98%) and artemisinin-d3 (C_15_H_19_D_3_O_5_, purity 98%) were of the internal standard (IS) and obtained from Toronto Research Chemicals Inc. (Toronto, Canada). High-performance liquid chromatography (HPLC)-grade acetonitrile and methanol were obtained from Merck Co. (Darmstadt, Germany). All other chemicals and reagents were of analytical grade and were procured from commercial sources.

### 2.2. Animals

The SD rats (7–8 weeks old, weighing 260–290 g (male) and 190–230 g (female)) were obtained from Guangdong Medical Laboratory Animal Center (Foshan, China), and Beagle dogs (8–9 months old, weighing 8–9 kg) were obtained from Nanjing Bigdoor Bioscience Inc. (Nanjing, China). The laboratory animal production license numbers were SCXK (Guangdong) 2018-0002 and SCXK (Suzhou) 2016-0007. Four rats were reared in a metal cage under standard laboratory conditions of room temperature (20–26°C) and relative humidity (40–70%). Dogs were housed in individual metal cages under temperatures ranging from 16°C to 26°C and relative humidity ranging from 40% to 70%. All animal experiments were conducted in compliance with the principles of good laboratory practice (GLP) from National Medical Products Administration (NMPA), China, and were performed in the laboratory animal room of New South Center of Safety Evaluation for Drugs of Guangzhou University of Chinese Medicine (Chinese animal use license number: SYXK (Guangdong) 2018-0014). Research protocols were approved by ethical committee for animal care and use based on 3R principal (reduction, replacement, and refinement).

### 2.3. Conditions for the Detection Method

The QTRAP™ 5500 LC/MS/MS system (AB SCIEX, Foster, CA, USA) including an autosampler, a dual pump, a column oven, and a triple tandem quadrupole mass detector was used to analyze the plasma samples. The chromatographic separation of hydroxychloroquine was achieved on a Synergi Fusion-RP C18 column (4 *μ*m, 150 × 2 mm, Phenomenex, Torrance, CA, USA) at 30°C. Water containing 0.6% formic acid and 5 mM ammonium acetate-methanol containing 0.6% formic acid (40 : 60, v/v) was used as the mobile phase at a flow rate of 0.4 mL/min. The separation of artemisinin was achieved on a Kinetex C18 column (2.6 *μ*m, 150 × 3 mm, Phenomenex, Torrance, CA, USA) at 30°C. The mobile phases consisted of 0.1% formic acid and 5 mM ammonium acetate in water-acetonitrile (15 : 85, v/v) at a flow rate of 0.5 mL/min, and the temperature of the autosampler was 4°C. Mass spectrometric detection was conducted with positive electrospray ionization in the multiple reaction monitoring (MRM) mode. The mass transitions were *m*/*z* 336.3 ⟶ 247.1 for hydroxychloroquine, *m*/*z* 340.3 ⟶ 251.2 for hydroxychloroquine-d4 (IS), *m*/*z* 300.4 ⟶ 209.1 for artemisinin, and *m*/*z* 303.3 ⟶ 212.3 for artemisinin-d3 (IS). The source temperature was maintained at 500°C, and the spray voltage was set at 5500 V. The nebulizer gas, heater gas, curtain gas, and collision-activated dissociation gas were nitrogen and set to 50, 50, 35, and medium, respectively. The data acquisition and analysis were controlled using the Analyst software™.

An aliquot of 10 *μ*L internal standard (hydroxychloroquine-d4 at 100 ng/mL) and 500 *μ*L of methanol containing 0.6% formic acid were added and was added to 10 *μ*L of rat or dog plasma samples, hydroxychloroquine standard samples, or QC samples. After vortex-mixing, the mixture was centrifuged at 12,000 rpm for 10 min at 4°C. An aliquot of 5 *μ*L supernatant was injected into the LC-MS/MS system to detect the concentration of hydroxychloroquine. Conventional liquid-liquid extraction was used to prepare artemisinin plasma samples. After 50 *μ*L of rat or dog plasma samples, artemisinin standard samples or QC samples were spiked with internal standard solution (artemisinin-d3 at 100 ng/mL), extraction was done with 600 *μ*L of ethyl acetate followed by centrifugation at 12,000 rpm for 5 min at 4°C. Next, an aliquot of the 500 *μ*L supernatant was collected and dried for 30 min using a RVC 2–25 CD plus vacuum centrifugal concentrator (CHRIST, Ostende, Germany), and dried residues were then redissolved in 100 *μ*L of water and acetonitrile (50 : 50, v/v) and centrifuged at 12,000 rpm for 5 min at 4°C. Finally, an aliquot of 10 *μ*L supernatant was loaded into the LC-MS/MS.

The methods were validated according to the US Food and Drug Administration (FDA) bioanalytical method validation guidance on selectivity, sensitivity, accuracy, precision, recovery, matrix effect, dilution effects, and stability under different conditions.

### 2.4. Animal Studies

AH was freshly prepared with 0.5% sodium carboxymethyl cellulose solution before administration to obtain a dose volume of 5 mL/kg body weight of animals for PK and TK studies in rats. The test article analysis of artemisinin and hydroxychloroquine sulfate in AH preparation (25–400 mg/mL) was performed before the initiation of the study, including concentration verification, homogeneity, and stability. The AH preparation was found to be even stable within 6 hours at room temperature (data not shown). The AH preparation on the day of the first or last administration was within 15% of the target concentration.

Eighteen SD rats of both genders, randomly divided into 3 groups, were treated with a single oral administration of AH preparation at a dose of 191, 382, and 764 mg/kg, respectively. Approximately, 300 *μ*L of blood samples were collected from jugular vein at predose and 5 min, 15 min, 30 min, 1 h, 1.5 h, 2 h, 4 h, 6 h, 8 h, 12 h, 24 h, and 48 h after dosing. Six Beagle dogs of both genders received three rounds of single oral administration of AH. The dosages were 53.8, 107.6, and 215.2 mg/kg, and the cleaning period was one week for each round. Approximately 1 mL of blood samples were collected from the forelimb vein at predose and 5 min, 15 min, 30 min, 1 h, 1.5 h, 2 h, 3 h, 4 h, 6 h, 8 h, 12 h, 24 h, 48 h, and 72 h after dosing. The TK studies in rats and dogs were accompanied by the 14-day repeated dosing studies. Four groups of eight SD rats of both genders, as satellite group, were given oral administration of AH preparation once daily at 146, 219, 328, and 492 mg/kg, respectively. Three groups of ten Beagle dogs each with equal gender ratio were administered orally once daily with AH at 56, 84, and 126 mg/kg. On day 1 (first administration) and day 14 (last administration), rat or dog blood samples were collected at predose and 10 min, 30 min, 1 h, 1.5 h, 2 h, 4 h, 6 h, 8 h, 12 h, and 24 h after dosing. All the above blood samples were collected in EDTA tubes, mixed by inversion, and placed on ice, and then centrifuged at 3000 rpm for 10 min at 4°C. The obtained plasma samples were stored at −80°C until analysis.

### 2.5. Kinetic Analysis

The PK and TK parameters were calculated from the plasma concentrations of the analytes versus time data using the noncompartmental analysis model of Drug and Statistics (DAS) software (version 3.2.8, BioGuider Co., Shanghai, China), including the area under the blood concentration curve from time zero to the last quantifiable time point or infinite time (AUC_0−*t*,_ AUC_0−∞_), elimination half-life (*t*_1/2_), mean residence time (MRT), apparent volume of distribution (Vd), and clearance (CL). The maximum blood concentration (*C*_max_) and the time to reach the maximum concentration (*T*_max_) were directly obtained from the experimental data. The multidose linear correlation analysis of DAS software was applied to assess the linear relationship of the analytes in the dose interval in PK studies and use the multiple-dose accumulation analysis of DAS software to assess the accumulation of the analytes in TK studies.

### 2.6. Statistical Analysis

Data were expressed as mean and standard deviation (means ± SD) and analyzed by SPSS 19.0 statistical software. The two-sided *t*-test was used to evaluate dose or gender differences in the kinetic parameters, and the paired-sample *t*-test was used to evaluate differences between the first and last doses in the kinetic parameters. Differences were considered significant when *P* ≤ 0.05.

## 3. Results

### 3.1. Method Validation Study

Typical chromatograms of rat blank plasma, blank plasma spiked with hydroxychloroquine or artemisinin, and the IS and dosed rat plasma samples are presented in Figure 1, and there is no significant interference from endogenous components at the retention times of hydroxychloroquine (0.73 min) and artemisinin (1.70 min). Good linear calibration curves were obtained over the concentration range from 1 ng/mL to 1000 ng/mL for both analytes, and the typical regression equations of the calibration curve were *y* = 1.08*x* + 0.00704 (regression coefficient (*r*) = 0.9986) for hydroxychloroquine and *y* = 4.28*x* + 0.00397 (*r* = 0.9996) for artemisinin, where *y* is the ratio of the analyte peak area to IS and *x* represents the plasma concentration of the analyte (weighting factor 1/*x*^2^). The accuracy and precision of the methods were validated by the analysis of the lower limit of quantification (LLOQ), low, mid, sub-high, and high plasma samples at five concentration levels (1, 2, 80, 400, 800 ng/mL) with six replicates in three analytical runs, and the results are summarized in Table 1. The intra- and inter-run precision values (RSD) of both analytes were less than 15%, while the accuracy values (RE) were within ±20%. The matrix effect was evaluated by comparing the peak area in the presence of matrix (measured by analyzing blank matrix spiked after extraction with analyte) to the peak area in the absence of matrix (pure solution of the analyte). The coefficient of variation (CV) of the IS-normalized matrix factor (MF) of both analytes calculated from the 6 lots of matrix was less than 15% at low and at high level of concentration. Standards as high as 4000 ng/mL in plasma could successfully be diluted 10-fold with observed acceptable accuracy and precision (hydroxychloroquine: RE 9.7%, RSD 7.8%; artemisinin: RE 3.7%, RSD 2.4%). Both analytes at low and high concentration levels in rat plasma were found to be stable after the exposure at 4°C for 4 h, in the autosampler at 4°C for 24 h, three freeze and thaw cycles and storage at −80°C for 60 days, and the accuracy of nominal concentrations were ranged from −11.2% to 10.5%. The methods were applied to the determination of the analyte concentration in dog plasma, only partial validation has been done, including a run of precision and accuracy, matrix effect, stability, and the results meet the criteria.

### 3.2. Pharmacokinetic Study

Mean plasma concentration versus time curves of hydroxychloroquine and artemisinin in rats are shown in Figure 2, and their PK parameters for the 3 doses are listed in Table 2. After a single oral administration of low, medium, and high doses of AH in rats, hydroxychloroquine was detectable from 5 min to 48 h; the plasma concentration gradually increased and reached maximum peak at 4–6 h (*T*_max_) and then cleared slowly from plasma with *t*_1/2_ of 10–15 h. There was no apparent gender difference in major PK parameters of hydroxychloroquine in rats (*P* > 0.05). The ratio of the average AUC_0−*t*_ of hydroxychloroquine among doses (1 : 1.96 : 3.98) was consistent with the relative dose ratio (1 : 2 : 4), whereas *C*_max_ (ratio 1 : 1.55 : 2.16) increased lower than proportionally to the dose. The result of multidose linear correlation analysis by DAS software confirmed that AUC showed a linear correlation with the dosage, while *C*_max_ was nonlinear.

Artemisinin was quickly absorbed into the blood following oral administration with *C*_max_ reaching at 5 min–1 h, followed by rapid clearing from plasma with *t*_1/2_ of 0.7–2 h; artemisinin was undetectable at 6 h in male rats and was detectable in female rats in low-, medium-, and high-dose groups at close to or lower than LLOQ at 6 h, 8 h, and 12 h, respectively. Compared with female rats, the AUC and *C*_max_ of artemisinin in male rats of low-, medium-, and high-dosing groups were significantly lower (*P* ≤ 0.05), and Vd and CL were significantly higher (*P* ≤ 0.05), which indicated that there were obvious gender differences in the pharmacokinetic profile of artemisinin in rats. The plasma concentration and exposure of artemisinin in female rats were ≥10-fold higher, and the clearance rate was lower than the male rats. In females, AUC_0−*t*_ of artemisinin showed a positive correlation with the dosage as the ratio of the average AUC_0−*t*_ (1 : 1.61 : 3.18) was close to the relative dose ratio (1 : 2 : 4), but *C*_max_ was not linearly related to the dose (ratio 1 : 1.49 : 1.90). In addition, there was no linear relationship between AUC_0−*t*_ or *C*_max_ and the dose level in males. The same was observed in the multidose linear correlation analysis results by DAS software.

As shown in Table 3, the apparent interindividual variability was observed in the pharmacokinetic parameters (AUC, *C*_max_, CL, etc.) of artemisinin in male and female rats (RSD > 40%), and the difference in males was larger, while that can also be seen in plasma concentration-time curves (based on % standard deviation) within each dose group. Except for *C*_max_ and *T*_max_, the interindividual variabilities in pharmacokinetic parameters of hydroxychloroquine were generally mild in rats.

The pharmacokinetic profile of hydroxychloroquine in dogs was similar to that in rats. In male and female dogs, following oral administration at three dose levels, hydroxychloroquine was detectable at all time points and was maintained at a high level from 2 h to 8 h, followed by a slow elimination phase (Figure 3). The results of PK parameters in dogs are given in Table 4. No apparent gender-related difference was found in the three dosages. The exposure of hydroxychloroquine with regard to AUC_0−*t*_ and *C*_max_ showed a linear correlation with the dosage as a relative dose ratio of 1 : 2 : 4 led to a AUC_0−*t*_ ratio of 1 : 1.93 : 3.94 and a *C*_max_ of 1 : 1.91 : 3.8, and linear correlation analysis by DAS software also show that both were linearly correlated. The pharmacokinetic parameters of hydroxychloroquine in dogs have less interindividual variability apart from *C*_max_ and *T*_max_, which was consistent with the case in rats. Since the plasma concentration of artemisinin was below or close to the LLOQ in dogs at each dose, we neither draw a complete plasma concentration-time curve nor obtained its PK parameters.

### 3.3. Toxicokinetic Study

The mean concentration-time curves (Figure 4), AUC, and *C*_max_ (Table 5) revealed that the exposure of hydroxychloroquine in rats increased as the doses of AH increased from 146 to 492 mg/kg, both on the first day (day 1) and the last day (day 14). The mean AUC and *C*_max_ of hydroxychloroquine in dogs, regardless of dose, increased on day 14 in comparison with day 1, and the difference of AUC was statistically significant (*P* ≤ 0.05). According to the results of multiple-dose accumulation analysis by DAS software (Table 3), the accumulation coefficients of hydroxychloroquine with regard to AUC in rats orally treated with AH for 14 days at four doses level were 1.5, 1.9, 1.8, and 1.7, respectively. In addition, the accumulation coefficients of *C*_max_ is greater than 1.5 at the high-dose levels. Therefore, hydroxychloroquine has a tendency to accumulate in rats following 14-day repeated oral administration of AH at doses of 146, 219, 328, and 492 mg/kg. In contrast, compared with day 1, AUC and *C*_max_ of artemisinin in females remarkably decreased on day 14 (Table 5), indicating that the exposure of artemisinin was reduced in female rats with repeated administrations of AH. This was probably because artemisinin can induce its own metabolism and has the time-dependent kinetic characteristics (*C*_max_ and AUC decrease with the prolonged administration period). The exposure changes of artemisinin with regard to *C*_max_ and AUC in male rats with repeated administrations of AH were inconsistent with each dose, and the causes may involve the low plasma concentration and great interindividual variability.

Based on the results of the 14-day repeated dosing study of AH in rats, the clinical toxicity symptoms, involving shedding of hair, emaciation, and mental restlessness, were dose- and time-dependent. Hematology and blood biochemistry results showed varying degrees of dose-dependent damage to the blood system, liver, and kidney functions (unpublished data). Dose-related pathological lesions to the liver, kidney, and spleen were observed in 328 and 492 mg/kg dose group at the end of the treatment period, mainly manifested as lobular central liver hypertrophy, hepatocyte vacuolation, vacuolar degeneration of renal cortex, and aggregation of splenic red pulp foam cells. The no-observed-adverse-effect level (NOAEL) for AH in rats was considered to be 219 mg/kg, and the lowest-observed-adverse-effect level (LOAEL) was 328 mg/kg. The toxicokinetic results were basically consistent with the above results as plasma exposure of hydroxychloroquine and artemisinin is positively correlated with the dose, and hydroxychloroquine has an increase in systemic exposure and accumulation in rats following repeated doses of AH.

According to the mean concentration-time curves (Figure 5) and the results of corresponding toxicokinetic parameters including AUC and *C*_max_ (Table 6), the exposure of hydroxychloroquine in dogs increased in a linear correlation with increasing doses after the first (day 1) and last administration (day 14). The mean AUC of hydroxychloroquine on day 14 was significantly increased than that on day 1 at low, medium, and high doses (56, 84, and 126 mg/kg) (*P* ≤ 0.05), and its corresponding accumulation coefficients were 1.5, 1.3, and 1.4 (Table 6), respectively, suggesting there was a mild accumulation in dogs following repeated doses of AH. The above toxicokinetic results were basically consistent with the 14-day repeated dosing study of AH in dogs, including the fact that the toxicity symptoms involved, vomiting, loose stools, decreased activity, and anorexia, were dose- and time-dependent, and high dose could cause pathological damage of spleen, etc. (unpublished data). The NOAEL for AH in dogs was established at 56 mg/kg, and the LOAEL was 126 mg/kg. It was of note that in the repeated administration toxicity studies, the toxic reaction of rats was stronger than that of dogs at the equivalent dose, which may be due to the greater exposure of hydroxychloroquine in rats.

## 4. Discussion

In the present study, obvious gender differences in the pharmacokinetics and toxicokinetics of artemisinin were observed in SD rats with higher plasma exposure and lower clearance rate in female rats, which is similar to the previous pharmacokinetic studies of artemisinin in rats [11, 12]. Gender difference in the pharmacokinetics of artemisinins has been reported only in animals and malaria patients [13], while not in healthy adults [14]. The reason may be the species differences in composition and activity of cytochrome P450 (CYP450) isoenzymes of human beings and animals, as well as the specificity of substrates and products of CYP450 enzymes. The level of CYP450 enzymes in female rats is 10–30% lower than that in male rats. The main metabolic enzymes activated by artemisinin, such as CYP2B and CYP3A, have gender differences in rats [15]. In addition, the main pharmacokinetic and toxicokinetic parameters of artemisinin had apparent interindividual variability in male and female rats, and *C*_max_ and AUC were overlapped between doses. Previously, Zang et al. [16] reported that there was a large interindividual variability in artemisinin pharmacokinetic parameters in 14 healthy adult male subjects with a % CV of 43.5% (6.9–122.7%) for AUC_0−*t*._ It may be caused by the genetic polymorphism of the CYP450 enzymes, which leads to differences in drug metabolism rates among individuals [17].

After 14-day repeated oral administration of AH in rats, the plasma exposure of artemisinin *in vivo* was reduced with time-dependent kinetic profile, i.e., *C*_max_ and AUC decreased with the prolongation of the administration period. Xing et al. [1] demonstrated that after the oral administration of artemisinin in rats for 5 successive days, the AUC of females and males were decreased by 63.5% and 56.4% and the *C*_max_ was decreased by 66.8% and 55.8%, respectively. Furthermore, several previous studies reported that the pharmacokinetics showed obvious time-dependent characteristics in healthy volunteers and malaria patients after repeated oral or rectal administration, but the relevant pharmacokinetic parameters of volunteers two weeks after drug withdrawal were similar to the results on day 1, suggesting that artemisinin could induce its own metabolism, and this induction process is recoverable, which may be related to changes in the activity of metabolic enzymes [16, 18, 19].

There have been two early papers that applied radioimmunoassay to investigate the pharmacokinetics in dogs following artemisinin, but artemisinin was not detected in dog serum [20, 21]. Li et al. [22] reported that dogs received a high dose of artemisinin (1000 mg), which was determined by LC-MS/MS with high sensitivity (LLOQ: 2 ng/mL), but negligible amounts of the artemisinin were detected in dog plasma (lower than 30 ng/mL), indicating artemisinin is poorly absorbed and metabolized rapidly in dogs. Whereas in our study, Beagle dogs were given three doses of AH orally, and the corresponding dose of artemisinin was 12.4–45.8 mg/kg, the concentration of artemisinin in plasma samples was below or close to LLOQ (1 ng/mL), which was similar to those reported above. A potential explanation for this outcome may be that the composition and activity of CYP450 enzymes induced by artemisinin varies with species.

Although the AUC of hydroxychloroquine in rats and dogs was linearly correlated to the administered dose, *C*_max_ was nonlinear, and there was apparent interindividual variability in *C*_max_ and *T*_max_, which may be related to certain differences in the plasma concentration of hydroxychloroquine among individuals, and it has been reported that the plasma concentration of hydroxychloroquine in humans has obvious individual difference [7, 23, 24]. We presume that the reason for this difference may be the metabolism regulation of hydroxychloroquine *in vivo* by a variety of CYP450 enzymes, such as CYP2D6, 2C8, 3A4/5, and differences in individual metabolic enzymes could lead to different plasma concentrations of hydroxychloroquine [25–27].

Hydroxychloroquine sulfate, as another component of AH, has no gender differences in animal PK and TK studies; therefore, we combined the data of both male and female animals in the same group for analysis. In addition, the data of male and female rats and dogs in the 14-day repeated toxicity studies were analyzed separately, including body weight, hematology, blood biochemistry, organ coefficients, etc. There was no gender difference in the toxic effects in these studies, and the detailed results will be published in the near future. Since the artemisinin has low toxicity, the toxicity of animals in 14-day repeated toxicity studies may be mainly due to hydroxychloroquine as it is basically consistent with the exposure of hydroxychloroquine in plasma, and is also consistent with the toxic effects of hydroxychloroquine in clinical applications, which mainly involves skin, gastrointestinal tract, central nervous system, cardiovascular system, hematology, etc. [28, 29]. It was of note that the toxic reaction in rats was significantly stronger than that in dogs at the equivalent dose; one reason might be the greater exposure of hydroxychloroquine in rats. It is suggested that the plasma concentration of hydroxychloroquine is one of the concerns in the observation of adverse reactions when AH is used long term for immune diseases such as rheumatoid arthritis and systemic lupus erythematosus in the future. Overall, the information from our studies might be helpful for further studies on the pharmacological and toxicological research of AH and beneficial for its clinical application.

## 5. Conclusion

We developed and validated the LC-MS/MS methods to detect the plasma concentration of hydroxychloroquine and artemisinin in SD rats and Beagle dogs and successfully applied it to the pharmacokinetic and toxicokinetic studies of AH in a single and repeated doses following oral administration to rats and dogs.

## Figures and Tables

**Figure 1:** Representative chromatograms for hydroxychloroquine, artemisinin, and the internal standards in rat plasma: (a) blank plasma sample, (b) blank plasma sample spiked with the IS, (c) LLOQ sample spiked with the IS, and (d) rat plasma sample 1 h after the oral dose of AH.

**Figure 2:** Mean plasma concentration-time curves of hydroxychloroquine (a) and artemisinin (female (b) and male (c)) in rats after a single oral administration at low, medium, and high doses of AH (191, 382, and 764 mg/kg).

**Figure 3:** Mean plasma concentration-time curve of hydroxychloroquine in Beagle dogs after a single oral administration at low, medium, and high doses of AH (53.8, 107.6, and 215.2 mg/kg).

**Figure 4:** Mean plasma concentration-time curve of hydroxychloroquine (a) and artemisinin (female (b) and male (c)) in rats after oral administration of AH at doses of 146, 219, 328, and 492 mg/kg on day 1 and day 14 during the course of the repeated dose TK study.

**Figure 5:** Mean plasma concentration-time curve of hydroxychloroquine in dogs after oral administration at low, medium, and high doses of AH (56, 84, and 126 mg/kg) on day 1 and day 14 during the course of the repeated dose TK study.

**Table 1:** Intra- and inter-run precision and accuracy of the method.

Analyte	Concentration (ng/mL)	Precision (RSD, %)				Accuracy (RE, %)			
		Intrarun			Inter-run	Intrarun			Inter-run
		Run 1	Run 2	Run 3		Run 1	Run 2	Run 3	
Hydroxychloroquine	1	13.5	3.8	5.2	7.5	−0.5	−3.1	−4.4	−2.7
	2	4.4	7.7	2.4	4.8	3.6	−13.0	−14.8	−8.1
	80	1.9	4.1	3.7	3.2	14.2	6.0	0.2	6.8
	400	2.7	4.0	2.4	3.1	−8.3	5.8	4.6	0.7
	800	4.2	2.5	2.6	3.1	13.9	−1.5	−1.4	3.7

Artemisinin	1	13.8	3.5	4.1	7.1	6.1	1.7	1.3	3.1
	2	9.0	4.8	8.0	7.3	−3.8	1.6	−0.2	−0.8
	80	4.6	2.4	3.5	3.5	−10.1	−2.6	−13.4	−8.7
	400	2.8	2.8	4.0	3.2	−8.8	−0.2	0.8	−2.7
	800	3.5	2.4	2.4	2.8	−8.1	−3.4	−4.3	−5.3

**Table 2:** Pharmacokinetic parameters of hydroxychloroquine and artemisinin in rats after oral administration.

Parameters	Hydroxychloroquine			Artemisinin					
				Female			Male		
	Low-dose	Mid-dose	High-dose	Low-dose	Mid-dose	High-dose	Low-dose	Mid-dose	High-dose
*C*_max_ (ng/mL)	402.6 ± 131.7	623.4 ± 114.0^*∗*^	868.5 ± 261.6^*∗*Δ^	357.3 ± 259.3	534.0 ± 236.5	679.0 ± 570.6	35.0 ± 27.5	69.8 ± 71.2^#^	46.2 ± 33.4
*T*_max_ (h)	3.9 ± 1.6	5.0 ± 1.1	5.8 ± 3.2	0.63 ± 0.60	0.50 ± 0.35	0.69 ± 0.38	0.63 ± 0.60	0.33 ± 0.20	0.44 ± 0.38
*t*_1/2_ (h)	9.7 ± 2.7	11.0 ± 2.0	14.8 ± 4.5^*∗*^	0.73 ± 0.14	0.69 ± 0.17	2.17 ± 1.92	1.30 ± 1.62	0.71 ± 0.47	1.55 ± 0.94
MRT_0−∞_ (h)	13.6 ± 2.9	16.2 ± 1.5	22.5 ± 5.3^*∗*Δ^	1.24 ± 0.19	1.41 ± 0.21	3.59 ± 1.87^*∗*^	1.97 ± 2.25	0.81 ± 0.38^#^	2.17 ± 1.64
Vd (mL/kg)	153.2 ± 80.3	160.3 ± 22.0	203.1 ± 43.6^△^	115.1 ± 43.0	151.9 ± 90.7	562.6 ± 669.4	4238 ± 6741	3378 ± 1706^#^	8314 ± 6234^#^
CL (mL/h/kg)	10.5 ± 2.4	10.2 ± 1.1	10.0 ± 2.8	112.9 ± 48.4	146.1 ± 65.9	148.2 ± 64.6	1564 ± 857^#^	4873 ± 3511	4356 ± 4032
AUC_0−*t*_ (h × ng/mL)	5006.8 ± 1020.4	9829.5 ± 940.7^*∗*^	19925.3 ± 4291.6^*∗*Δ^	407.1 ± 169.6	655.7 ± 308.0	1294.5 ± 797.0	30.2 ± 26.8^#^	43.4 ± 59.6^#^	44.0 ± 32.8^#^
AUC_0−∞_ (h × ng/mL)	5174.0 ± 966.7	10373.7 ± 1107.5^*∗*^	22419.7 ± 5599.7^*∗*Δ^	416.2 ± 177.0	658.7 ± 306.2	1335.8 ± 761.2	34.5 ± 23.0^#^	46.4 ± 63.6^#^	64.4 ± 43.4^#^

^∗^ *P* significant difference from low-dose, ^Δ^*P* ≤ 0.05 significant difference from mid-dose, and ^#^*P* ≤ 0.05 significant difference from female.

**Table 3:** Individual differences in pharmacokinetic parameters of hydroxychloroquine and artemisinin in rats.

Parameters	Hydroxychloroquine, precision (RSD, %)			Artemisinin, precision (RSD, %)					
				Female			Male		
	Low-dose	Mid-dose	High-dose	Low-dose	Mid-dose	High-dose	Low-dose	Mid-dose	High-dose
*C*_max_	32.7	18.3	30.1	72.6	44.3	84.0	78.6	102.1	72.3
*T*_max_	41.0	21.4	54.4	95.2	70.8	54.5	95.2	61.3	85.6
*t*_1/2_	28.1	17.8	30.3	18.6	23.9	88.6	123.9	66.9	60.8
MRT_0−∞_	21.6	9.6	23.7	15.4	15.0	52.0	114.1	47.0	75.7
Vd	52.4	13.7	21.5	37.4	59.7	119.0	159.1	50.5	75.0
CL	23.0	11.1	28.4	42.8	45.1	43.6	54.8	72.1	92.6
AUC_0−*t*_	20.4	9.6	21.5	41.6	47.0	61.6	88.8	137.2	74.6
AUC_0−∞_	18.7	10.7	25.0	42.5	46.5	57.0	66.9	137.1	67.4

**Table 4:** Pharmacokinetic parameters of hydroxychloroquine in dogs after oral administration.

Parameters	Low-dose	Mid-dose	High-dose
*C*_max_ (ng/mL)	269.0 ± 164.4	534.2 ± 241.1	1183.8 ± 352.5^*∗*Δ^
*T*_max_ (h)	1.4 ± 1.1	1.8 ± 0.8	2.9 ± 2.7
*t*_1/2_ (h)	25.4 ± 3.5	22.2 ± 6.8	21.4 ± 8.0
MRT_0−∞_ (h)	33.9 ± 4.8	29.5 ± 9.4	26.7 ± 8.0
Vd (mL/kg)	123.8 ± 19.1	109.9 ± 22.7	108.8 ± 45.7
CL (mL/h/kg)	3.4 ± 0.8	3.5 ± 0.6	3.5 ± 0.5
AUC_0−*t*_ (h × ng/mL)	3970.4 ± 821.4	7681.9 ± 1147.5^*∗*^	15644.0 ± 2610.2^*∗*Δ^
AUC_0−∞_ (h × ng/mL)	4492.5 ± 1042.7	8593.0 ± 1520.3^*∗*^	17078.6 ± 2875.9^*∗*Δ^

^*∗*^ *P* ≤ 0.05 significant difference from low-dose and ^Δ^*P* ≤ 0.05 significant difference from mid-dose.

**Table 5:** Toxicokinetic parameters of hydroxychloroquine and artemisinin in rats after oral administration.

Analyte	Gender	Doses (mg/kg)	*C*_max_ (ng/mL)		AUC_0−*t*_ (h × ng/mL)		Accumulation coefficient of *C*_max_	Accumulation coefficient of AUC
			Day 1	Day 14	Day 1	Day 14		
Hydroxychloroquine	Female + male	46	308.5 ± 87.7	346.0 ± 179.8	2859.0 ± 656.2	4274.9 ± 1083.2^*∗*^	1.1	1.5
		219	616.7 ± 521.8	590.4 ± 169.6	4284.0 ± 916.1	7749.1 ± 1826.0^*∗*^	1.3	1.9
		328	400.3 ± 155.8	631.5 ± 104.4^*∗*^	5408.3 ± 1463.5	9287.9 ± 1279.7^*∗*^	1.8	1.8
		492	565.6 ± 301.6	826.0 ± 253.7^*∗*^	7086.1 ± 1718.3	11660.3 ± 2242.7^*∗*^	1.6	1.7

Artemisinin	Female	46	154.8 ± 119.1	46.9 ± 24.3	161.6 ± 86.8	83.8 ± 37.6	0.4	0.6
		219	319.3 ± 97.3	150.8 ± 218.6	369.3 ± 104.4	138.4 ± 89.2	0.5	0.4
		328	341.5 ± 293.7	38.1 ± 17.3	451.9 ± 434.2	85.7 ± 26.0	0.3	0.6
		492	270.8 ± 128.1	84.2 ± 48.8^*∗*^	379.3 ± 370.8	224.9 ± 110.1	0.3	0.8
	Male	46	2.8 ± 2.4	7.1 ± 2.1	2.9 ± 2.4	15.1 ± 4.0	1.8	2.5
		219	12.7 ± 5.5	12.3 ± 4.5	10.1 ± 4.0	25.0 ± 11.6	1.1	2.9
		328	10.9 ± 5.0	7.5 ± 4.9	21.2 ± 10.8	12.2 ± 9.3	0.8	0.7
		492	39.3 ± 54.3	23.3 ± 22.9	37.7 ± 23.7	19.4 ± 11.0	2.3	0.6

^*∗*^ *P* ≤ 0.05 significant difference from day 1.

**Table 6:** Toxicokinetic parameters of hydroxychloroquine in dogs after oral administration.

Parameters	Low-dose		Mid-dose		High-dose	
	Day 1	Day 14	Day 1	Day 14	Day 1	Day 14
*C*_max_ (ng/mL)	222.4 ± 68.7	293.7 ± 97.4	454.0 ± 122.2	440.4 ± 161.5	597.0 ± 335.0	490.6 ± 118.4
AUC_0−*t*_ (h × ng/mL)	2129.9 ± 586.0	3272.5 ± 1258.4^*∗*^	3988.5 ± 783.0	5208.6 ± 1667.8^*∗*^	5722.4 ± 1554.0	7118.6 ± 1294.9^*∗*^
Accumulation coefficient of *C*_max_	1.5		1.0		1.1	
Accumulation coefficient of AUC	1.5		1.3		1.4	

^*∗*^ *P* ≤ 0.05 significant difference from day 1.

## Data Availability

The data used to support the findings of this study are available from the corresponding author upon request.

## References

[1] World Health Organization (2020). *World Malaria Report 2020: 20 Years of Global Progress and Challenges*.

[2] Menard D., Dondorp A. (2017). Antimalarial drug resistance: a threat to malaria elimination. *Cold Spring Harbor Perspectives in Medicine*.

[3] Han C. M. (1978). Studies on the occurrence of a strain of chloroquine-resistant Plasmodium falciparum in Papua New Guinea. *PNG Medical Journal*.

[4] Muller O., Lu G. Y., von Seidlein L. (2019). Geographic expansion of artemisinin resistance. *Journal of Travel Medicine*.

[5] van der Pluijm R. W., Imwong M., Chau N. H. (2019). Determinants of dihydroartemisinin-piperaquine treatment failure in Plasmodium falciparum malaria in Cambodia, Thailand, and Vietnam: a prospective clinical, pharmacological, and genetic study. *The Lancet Infectious Diseases*.

[6] Ben-Zvi I., Kivity S., Langevitz P., Shoenfeld Y. (2012). Hydroxychloroquine: from malaria to autoimmunity. *Clinical Reviews in Allergy and Immunology*.

[7] Al-Bari M. A. (2015). Chloroquine analogues in drug discovery: new directions of uses, mechanisms of actions and toxic manifestations from malaria to multifarious diseases. *Journal of Antimicrobial Chemotherapy*.

[8] Salako L. A. (1984). Toxicity and side-effects of antimalarials in Africa: a critical review. *Bulletin of the World Health Organization*.

[9] Jorge A., Ung C., Young L. H., Melles R. B., Choi H. K. (2018). Hydroxychloroquine retinopathy - implications of research advances for rheumatology care. *Nature Reviews Rheumatology*.

[10] Hu C., Lu L., Wan J. P., Wen C. (2017). The pharmacological mechanisms and therapeutic activities of hydroxychloroquine in rheumatic and related diseases. *Current Medicinal Chemistry*.

[11] Xing J., Du F. Y., Liu T., Zhu F. P. (2012). Autoinduction of phase I and phase II metabolism of artemisinin in rats. *Xenobiotica*.

[12] Ashton M., Johansson L., Thornqvist A. S., Svensson U. S. (1999). Quantitative in vivo and in vitro sex differences in artemisinin metabolism in rat. *Xenobiotica*.

[13] Simpson J. A., Agbenyega T., Barnes K. I. (2006). Population pharmacokinetics of artesunate and dihydroartemisinin following intra-rectal dosing of artesunate in malaria patients. *PLoS Medicine*.

[14] Hong X., Liu C. H., Huang X. T. (2008). Pharmacokinetics of dihydroartemisinin in Artekin tablets for single and repeated dosing in Chinese healthy volunteers. *Biopharmaceutics and Drug Disposition*.

[15] Martignoni M., Groothuis G. M., de Kanter R. (2006). Species differences between mouse, rat, dog, monkey and human CYP-mediated drug metabolism, inhibition and induction. *Expert Opinion on Drug Metabolism and Toxicology*.

[16] Zang M., Zhu F., Li X., Yang A., Xing J. (2014). Auto-induction of phase I and phase II metabolism of artemisinin in healthy Chinese subjects after oral administration of a new artemisinin-piperaquine fixed combination. *Malaria Journal*.

[17] Zhou S. F., Liu J. P., Chowbay B. (2009). Polymorphism of human cytochrome P450 enzymes and its clinical impact. *Drug Metabolism Reviews*.

[18] Gupta S., Svensson U. S., Ashton M. (2001). In vitro evidence for auto-induction of artemisinin metabolism in the rat. *European Journal of Drug Metabolism and Pharmacokinetics*.

[19] Zhang S. Q., Hai T. N., Ilett K. F., Huong D. X., Davis T. M., Ashton M. (2001). Multiple dose study of interactions between artesunate and artemisinin in healthy volunteers. *British Journal of Clinical Pharmacology*.

[20] Zhao K., Chen Q., Song Z. (1986). Studies on the pharmacokinetice of qinghaosu and two of its active derivatives in dogs. *Acta Pharmaceutica Sinica*.

[21] Zhao K., Song Z. (1990). The pharmacokinetics of dihydroqinghaosu given orally to rabbits and dogs. *Acta Pharmaceutica Sinica*.

[22] Li C., Wang R., Zhang L., Zhang S. (2011). Determination of artemisinin in dog plasma by LC-MS/MS. *Chinese Remedies and Clinics*.

[23] Carmichael S. J., Day R. O., Tett S. E. (2013). A cross-sectional study of hydroxychloroquine concentrations and effects in people with systemic lupus erythematosus. *Internal Medicine Journal*.

[24] Furst D.E. (1996). Pharmacokinetics of hydroxychloroquine and chloroquine during treatment of rheumatic diseases. *Lupus*.

[25] Kim K. A., Park J. Y., Lee J. S., Lim S. (2003). Cytochrome P450 2C8 and CYP3A4/5 are involved in chloroquine metabolism in human liver microsomes. *Archives of Pharmacal Research*.

[26] Gil J. P., Gil Berglund E. (2007). CYP2C8 and antimalaria drug efficacy. *Pharmacogenomics*.

[27] Marki-Zay J., Tauberne Jakab K., Szeremy P., Krajcsi P. (2013). MDR-ABC transporters: biomarkers in rheumatoid arthritis. *Clinical and Experimental Rheumatology*.

[28] Lebin J. A., LeSaint K. T. (2020). Brief review of chloroquine and hydroxychloroquine toxicity and management. *Western Journal of Emergency Medicine*.

[29] Alanagreh L., Alzoughool F., Atoum M. J. A. (2020). Risk of using hydroxychloroquine as a treatment of COVID-19. *The International Journal of Risk and Safety in Medicine*.

